The article "The Influence of Walking Height and Width on the Gait" was published in 2021. Journal: J Healthc Eng.

# The Influence of Walking Height and Width on the Gait

**DOI:** 10.1155/2021/6675809

**Published:** 2021-06-23

**Authors:** Heng Ma, Yuanwen Min, Fangfang Wu, Xianglin Gao, Xiujuan Ma, Jie Yao, Chao Ma, Xiaoliu Li

**Affiliations:** ^1^Zhejiang Huadian Equipment Testing Institute (Zhejiang Key Laboratory for Protection Technology of High-Rise Operation), Hangzhou, Zhejiang, China; ^2^Key Laboratory for Biomechanics and Mechanobiology of Ministry of Education, School of Biological Science and Medical Engineering, Beijing Advanced Innovation Centre for Biomedical Engineering, Beihang University, Beijing, China; ^3^Key Laboratory of Modern Measurement and Control Technology (Ministry of Education), Beijing Information Science and Technology University, Beijing, China; ^4^Department of Rehabilitation, Minhang Hospital, Fudan University, Shanghai, China

## Abstract

Walking stability is an important factor that is related to working accidents at height. The understanding of the relationship between walking stability and walking conditions remains an unmet need. Therefore, this study aimed to investigate the effect of path height, width, and asymmetric conditions on the pressure and time information of the foot-ground interaction during walking. 12 subjects were required to walk at two height, three width, and asymmetric conditions. Plantar pressures during walking were measured with the F-scan insole sensors. The total pressures were normalized with body weight, and the temporal parameters were normalized with stance time. When the walking height increased, the plantar pressure at the “heel strike” phase did not change significantly, while that at “heel rise” and “toe off” phases significantly increased, and the “heel rise” occurred earlier, indicating a greater foot-ground interaction at the forefoot part of the sole. As the path width increased from 0.6 m to 1.2 m, the foot-ground interaction as well as the asymmetric effect approached to that of overground walking. The findings could help improve the risk assessment and footwear design.

## 1. Introduction

Working at height is one of the biggest causes of fatalities and major injuries. Fall from a height is the major accident type [1–3]. The spinal and head fractures can lead to severe disability or even death [4–9]. The recurrent mistake rate may even increase in people with accident experience. The regulation and funding to prevent falls from height have been evolving over the years; devices and trainings of fall prevention have been improved. However, the rate of accidental fall deaths remains high [10, 11].

Fall caused by the loss of balance is the most common accident during working at height [12–15]. The imbalance at height is caused by many factors including complicated neuromotor effects [16, 17]. Unstable and trembling behavior could be observed at height or virtual height [18–20], which could be amplified by environmental loads. It was reported that gait and balance ability can be improved through high-platform training [21, 22], but the mechanism was not clarified. It is important to explore the relation of gait and balance ability during working at height, through which valuable information for improving prevention strategies can be provided.

The article "The Influence of Walking Height and Width on the Gait" was published in 2021. Journal: J Healthc Eng.

As a typical activity of working at height, walking is closely related to the balance ability of people [23–25]. Gait analysis has been applied to study the impact of the high-altitude working condition on balance ability. There is ample evidence for pathway height and width associated with posture control during walking. It has been reported that higher pathway can lead to changes in joint kinematics and muscle activation on account of psychological factors [26, 27]. The heights investigated in the above studies were lower than 1.0 m, which is far lower than the realistic condition of working at height. Simeonov used virtual reality (VR) technology to simulate walking on a roof plank and observed the effect of height on the lateral angular velocities of the trunk and rearfoot [28]. Motion sickness caused by VR technology could be confused with the effect of path height and width on walking [29, 30]. The effects of narrow and wide path width on the trunk and joint kinematics have been compared [27, 28, 31]. Yet, how does the high-platform walking approaches to the ground walking with increasing the path width remains unclear, which is useful for the optimal configuration of path width for working at height. Besides, few studies have considered the asymmetric condition of pathway on walking at height, while asymmetric condition is common in working at height, such as working at the edge of the roof.

Apart from the need to assess the risk factors of height and width for walking at height, it was noticed that footwear design could affect the walking stability. Studies on older people have revealed the significant effect of the footwear interface on the posture stability in terms of plantar pressure [32, 33]. A study compared the trunk and foot kinematics when walking with different types of shoes at height [28]. However, the changes in plantar pressure during walking at height remain unclear, which could be important data for footwear optimization.

In this light, this study aimed to investigate the plantar pressure in different walking height, width, and asymmetric conditions. A platform of 10 m in height was used to simulate the environment of working at height. The plantar pressure and phase parameters were measured in three different path widths (0.6 m, 0.9 m, and 1.2 m). In addition, the high platform was designed to be unilateral dangerous condition, and plantar pressures during walking in the dangerous and safe sides were compared. The study can provide a better understanding of the interaction between walking conditions and the gait pattern and help improve the risk assessment and footwear design.

The article "The Influence of Walking Height and Width on the Gait" was published in 2021. Journal: J Healthc Eng.

## 2. Methods

### 2.1. Participants

Twelve healthy university students (six males and six females) voluntarily participated in the experiment. The mean ± SD for age, height, and body mass was 22.4 ± 0.8 years, 1.69 ± 4.8 m, and 62.6 ± 10.3 kg, respectively. The participants were excluded if they had any history of musculoskeletal diseases, cardiovascular and cerebrovascular diseases, acrophobia, neurological disorders, or visual abnormalities. The subjects were required to refrain from alcohol and not to participate in the competitive sports for at least one week before the experiment. The subjects were asked to walk on the high platform for 15 minutes every day to familiarize themselves with the trials since three days before the experiment. The study was approved by the Ethics Review Board of Beihang University. Every participant received an oral and written explanation of the study and signed inform consent before performing the trials.

### 2.2. Procedure

In this experiment, the F-scan plantar pressure measurement system (Tekscan Inc., Boston, MA, USA) was used to collect the plantar pressure information during walking with a sampling frequency of 50 Hz. The pressure sensors (size of 2.5*∗*2.5 mm^2^) were evenly distributed on the F-scan insole (3.9 sensors per square centimeter) (Figure 1). The F-scan insoles could be trimmed to fit the subject's footwear. To eliminate the side effect of footwear type, subjects were required to wear the same type of sneakers with proper sizes. The F-scan insoles were calibrated according to the body weight of the subject before each trial. The plantar pressure data during the experiment were transmitted to the computer wirelessly.

In the control group, subjects were required to walk straightly at self-selected walking speeds on the ground. In the experiment group, subjects were required to walk on a 10 m-high platform (Figure 2). Three different path widths (0.6 m, 0.9 m, and 1.2 m) were tested to investigate the effect of path width on the foot-ground interaction during walking at height. Since the realistic walking environment for working at height is usually asymmetric, the asymmetric path with one side dangerous and the other safe was used in this study. For each trial, the plantar pressure data were recorded after three minutes of warming up. Six full gait cycles in the middle of the trial were extracted for analysis. The gait cycle started when one foot contacted the ground and ended when that same foot contacted the ground again. The first and last gait cycles were ignored to eliminate the walking acceleration and deceleration effects [34]. Each trail lasted for four minutes and was repeated four times with three-minute intervals.

The article "The Influence of Walking Height and Width on the Gait" was published in 2021. Journal: J Healthc Eng.

### 2.3. Data Processing and Statistical Analysis

Each gait cycle was divided into the stance phase and swing phase. The total pressure was normalized with the body weight. Since the pressure was only nonzero during the stance phase, the temporal information of the pressure was normalized with stance phase time.

Statistical analysis was performed with SPSS 21.0 (SPSS Inc., Chicago, IL, USA). The F-test was used to verify homogeneity of variance, and then one-way ANOVA was used to analyze the influence of the height, width, and asymmetric condition on the foot-ground interaction.

## 3. Results

### 3.1. The Effect of Height on the Foot-Ground Interaction

The changes in total plantar pressure are shown in Figure 3(a). The maximum pressures occurred at “heel strike” and “toe off” during both ground and high-platform walking, and the minimum pressure occurred at “heel rise.” Compared with the ground walking, the total pressure of high-platform walking was similar at “heel strike” (no significant difference), whereas it was significantly greater at “heel rise” (*p* < 0.001) and “toe off” (*p*=0.023) (Figure 3(b)).

In terms of temporal characteristics, “heel strike” and “toe off” occurred approximately simultaneously at both high-platform walking (20.58 ± 3.31% and 79.61 ± 2.88% of the stance phase) and ground walking (20.18 ± 2.40% and 79.85 ± 3.05%), yet “heel rise” of high-platform walking (45.12 ± 6.41%) occurred significantly earlier than that of ground walking (47.50 ± 5.49%) (*p*=0.007).

### 3.2. The Effect of Walking Path Width on the Foot-Ground Interaction

The effect of path width on plantar pressure is shown in Figure 4(a). At “heel strike,” there were no significant differences between ground walking and high-platform walking with varying path width. Yet, at “heel rise” and “toe off,” with increasing path width, the plantar pressure during high-platform walking approached to that of ground walking. In particular, at “heel rise,” the plantar pressure of 0.6 m width was significantly greater than that of 0.9 m width (*p*=0.028), 1.2 m width (*p*=0.028), and ground walking (*p* < 0.001). The plantar pressure of 0.9 m width was also significantly greater than that of ground walking (*p*=0.05). Yet, there was no significant difference between ground walking and high-platform walking with 1.2 m path width. At “toe off,” the plantar pressures of 0.6 m and 0.9 m widths were significantly greater than those of ground walking (*p*=0.043 and 0.005, respectively), yet there was still no significant difference between ground walking and high-platform walking with 1.2 m path width. In terms of temporal characteristics (Figure 4(b)), “heel rise” of high-platform walking with 0.6 m and 0.9 m path widths (20.58 ± 3.31% and 21.13 ± 3.81% of the stance phase) occurred significantly earlier than that of ground walking (20.18 ± 2.40%) (*p*=0.007 and 0.029, respectively). Yet, there was no significant difference between ground walking and high-platform walking with 120 cm path width.

The article "The Influence of Walking Height and Width on the Gait" was published in 2021. Journal: J Healthc Eng.

### 3.3. The Effects of the Asymmetric Condition on the Foot-Ground Interaction

No significant differences were observed between the plantar pressures of dangerous and safe sides.  Figure 5 shows the effect of the asymmetric condition on heel rise time of high-platform walking. With 0.6 m and 0.9 m path widths, “heel rise” of the dangerous side occurred significantly earlier than that of ground walking (*p* < 0.05), while “heel rise” of the safe side had no significant difference with ground walking. No significant differences between dangerous and safe sides at “heel strike” and “toe off” phases were observed.

## 4. Discussion

The height and width of the path are major factors that influence the gait pattern during working at height, which is closely related to the risk of fall accidents. Few studies have measured the gait parameters in realistic walking at height (Table 1). VR technology has been used to simulate the walking condition at height [28]. However, motion sickness caused by VR may interfere with the accuracy of the experimental results. In this study, the impact of realistic asymmetric high-platform walking on plantar pressure was quantified. The plantar pressure significantly increased at heel rise and toe off phases and gradually decreased to that of ground walking with increasing the path width. The findings could provide knowledge for the risk assessment and environment optimization for working at height.

### 4.1. Effect of Height on the Gait

During walking, the plantar pressure experienced a maximum at the “heel strike” phase, a minimum at the “heel rise” phase, and the second maximum at the “toe off” phase. When the path height increased, the plantar pressure at “heel strike” did not change significantly, while that at “heel rise” significantly increased, and the “heel rise” occurred significantly earlier. The findings imply that subjects shifted their weight to the other foot faster and more intensely when walking at height. A similar phenomenon has been observed in Simeonov's study [28]. The angular velocity and lateral angular velocity of the rearfoot at the midstance phase increased with the walking height. Previous studies also reported no significant difference of the tibialis anterior muscle (activated during the heel strike phase in gait) between ground and high-platform walking [26, 27], which coincides with our results of plantar pressure at the “heel strike” phase. Furthermore, we found that “heel rise” occurred earlier during height walking, while the toe off did not, which implies a longer double-support time [26]. Unlike the simulated or simplified height condition in previous studies, this study was conducted based on a high-platform experiment. The greater plantar pressure during “heel rise” and “toe off” means that the interaction between the forefoot and the ground plays an important role in the balance during walking at height. Hence, the insole and outsole material of shoes should be more pliable with better stability in the forefoot part.

The article "The Influence of Walking Height and Width on the Gait" was published in 2021. Journal: J Healthc Eng.

### 4.2. Effect of Width on the Gait

The gait pattern was also significantly affected by the path width of walking at height according to our results. Considering the experiment safety, the path width was set to be 0.6 m, 0.9 m, and 1.2 m. In the 0.6 m-width and 0.9 m-width group, the plantar pressure at “heel rise” and “toe off” was greater than in the ground group; meanwhile, the “heel rise” phase also occurred earlier. In previous studies, paths with smaller width were applied.

The effect of width on foot lateral kinematics [28] and tibialis anterior muscle activation [27] was consistent with our results. The present study further showed that the influence of height on the gait pattern tends to be reduced along with the path width. The gait difference between the 1.2 m-width group and ground group was not significant according to our results, which should be fully considered in the optimal configuration of safe path width for working at height.

### 4.3. Effect of Asymmetry on the Gait

Gait symmetry is also a widely used index to assess fall risk [36, 37]. In this study, no significant difference was found between the plantar pressures at the dangerous and safe sides. Yet, the “heel rise” at the dangerous side occurred significantly earlier than that at ground walking, while “heel rise” at the safe side had no significant difference. The results implied that subjects tended to shift their weight from the dangerous side to the safe side. As the path width increased, the asymmetry disappears. In the previous studies of walking at height, the influence of asymmetry was not considered, yet the realistic working environment is often asymmetric, such as the edge of the roof or the scaffolding channel on the side of the building. The asymmetry factor should be concerned in the future studies and applications.

The article "The Influence of Walking Height and Width on the Gait" was published in 2021. Journal: J Healthc Eng.

There are some limitations in this study. Firstly, only the differences between the ground and 10 m-high platform were compared. The influence of different heights on the gait would be investigated in subsequent studies. Secondly, a unilateral dangerous condition was investigated in this study. For safety, it was not compared with the bilateral dangerous condition. Besides, unilateral dangerous condition is a typical condition for working at height such as the edge of the roof and the scaffolding channel on the side of the building. The present findings can provide a better understanding of the interaction between walking conditions and the gait pattern and help improve the risk assessment and footwear design.

The effect of height, width, and asymmetric conditions during height walking on gait parameters was quantified in this study. When the walking height increased, the plantar pressure at the “heel strike” phase did not change significantly, while that at “heel rise” and “toe off” phases significantly increased, and the “heel rise” occurred earlier, indicating a greater foot-ground interaction at the forefoot part of the sole. Asymmetry significantly affects the time of the “heel rise” phase. As the path width increased from 0.6 m to 1.2 m, the foot-ground interaction as well as the asymmetric effect approached to that of overground walking. The findings could help improve the risk assessment and footwear design.

## 5. Conclusion

When the walking height increased, the plantar pressure at the “heel strike” phase did not change significantly, while that at “heel rise” and “toe off” phases significantly increased, and the “heel rise” occurred earlier, indicating a greater foot-ground interaction at the forefoot part of the sole. Asymmetry significantly affects the time of the “heel rise” phase. As the path width increased from 0.6 m to 1.2 m, the foot-ground interaction as well as the asymmetric effect approached to that of overground walking. The findings could help improve the risk assessment and footwear design.

## Figures and Tables

**Figure 1:** Configuration of the F-scan plantar pressure measurement system. (a) F-scan insoles and sneakers. The pressure sensors were evenly distributed on the insoles. (b) Subject wearing the F-scan insoles and sneakers. The data collector obtains the plantar pressure data, and they are transmitted to the computer wirelessly.

The article "The Influence of Walking Height and Width on the Gait" was published in 2021. Journal: J Healthc Eng.

**Figure 2:** Diagram of walking conditions. Subjects were required to walk at a 10 m-high platform, with one side dangerous and the other safe. Three widths of the path were considered in the experiment.

**Figure 3:** Effect of walking height on plantar pressure. (a) Changes of average total plantar pressure in the stance phase of the gait cycle during ground walking and high-platform walking with 0.6 m width at the dangerous side. The maximum pressures occurred at “heel strike” and “toe off”; the minimum pressure occurred at “heel rise.” (b) Average total plantar pressure at “heel strike,” “heel rise,” and “toe off” phases. Plantar pressures of high-platform walking were significantly greater than those of ground walking at “heel rise” and “toe off.”

**Figure 4:** Effect of path width on pressure and temporal characteristics of the foot-ground interaction at the dangerous side. (a) At “heel rise” and “toe off” phases, the plantar pressures of high-platform walking with 0.6 m and 0.9 m path widths were significantly greater than those of ground walking. When path width was increased to 1.2 m, there was constantly no significant difference between ground walking and high-platform walking at all stance phases. (b) “Heel rise” of high-platform walking with 0.6 m and 0.9 m path width occurred significantly earlier than that of ground walking. There was no significant difference between the ground walking and high-platform walking with 120 cm path width.

**Figure 5:** Effect of the asymmetric condition on heel rise time. With 0.6 m and 0.9 m path widths, “heel rise” of the dangerous side occurred significantly earlier than that of ground walking, while “heel rise” of the safe side had no significant difference with ground walking. Yet, they did not present significant difference between each other.

**Table 1:** Studies on the influence of walking height and width on gait parameters.

Study	Subject	Walking conditions			VR	Gait parameters
		Height	Width	Other conditions		
Present study	Young people	Ground and 10 m	0.6 m, 0.9 m, and 1.2 m	Asymmetric	No	Plantar pressure and gait phase
Simeonov [28]	Construction workers	Virtual ground and roof plank	0.15 m and 0.25 m	Tilted floor, shoe style	Yes	Trunk and rearfoot lateral angular velocities
Delbaere [26]	Older people	Ground and 0.6 m	0.4 m	Bright and dim	No	Speed, step length, stride width, cadence, double-support time, EMG
Caballero [31]	Young people	Ground	0.15 m and 0.3 m	Ground stiffness, direction of a circular pathway	No	Sacral displacement and its mean velocity
Brown [27]	Younger and older adults	Ground and 0.6 m	0.15 m and 0.6 m	—	No	Joint kinematics and muscle activation
McAndrew Young and Dingwell [35]	Young healthy adults	Treadmill	Voluntary narrower, normal, and wider step widths	Metronome	No	Centre of mass motion

The article "The Influence of Walking Height and Width on the Gait" was published in 2021. Journal: J Healthc Eng.

## Data Availability

The data used to support the findings of this study are available from the corresponding author upon request.
